The article "Stability and Hopf Bifurcation Analysis of an Epidemic Model with Time Delay" was retracted in 2023. Reasons: signs of a paper mill; suspected computer-generated content; unreliable results or conclusions; concerns about the data.

# Stability and Hopf Bifurcation Analysis of an Epidemic Model with Time Delay

**DOI:** 10.1155/2021/1895764

**Published:** 2021-07-01

**Authors:** Yue Zhang, Xue Li, Xianghua Zhang, Guisheng Yin

**Affiliations:** ^1^College of Computer Science and Technology, Harbin Engineering University, Harbin 150001, China; ^2^School of Computer Science and Technology, Harbin Institute of Technology, Harbin 150001, China; ^3^College of Science, Heilongjiang University of Science and Technology, China

## Abstract

Epidemic models are normally used to describe the spread of infectious diseases. In this paper, we will discuss an epidemic model with time delay. Firstly, the existence of the positive fixed point is proven; and then, the stability and Hopf bifurcation are investigated by analyzing the distribution of the roots of the associated characteristic equations. Thirdly, the theory of normal form and manifold is used to drive an explicit algorithm for determining the direction of Hopf bifurcation and the stability of the bifurcation periodic solutions. Finally, some simulation results are carried out to validate our theoretic analysis.

## 1. Introduction

Today, the serious epidemics, such as SARS and H1N1, are still threatening the life of people continually. Plenty of mathematical models have been proposed to analyze the spread and the control of these diseases [1–7].

However, many infectious diseases, for instance, gonorrhea and syphilis, occur and spread amongst the mature, while some epidemics, for example, chickenpox and FMD, only result in infection and death in immature. For this reason, stage structure should be taken into consideration in models. Aliello and Freedman [8] proposed a stage-structured model described by

(1) $$\begin{array}{c} \left\{\begin{array}{c} \dot{x}\left(t\right)=\alpha y\left(t\right)-\gamma x\left(t\right)-\alpha e^{-\gamma \tau }y\left(t-\tau \right)\\ \dot{y}\left(t\right)=\alpha e^{-\gamma \tau }y\left(t-\tau \right)-\beta y^{2}\left(t\right) \end{array}\right., \end{array}$$

where *x*(*t*) is the immature population density and *y*(*t*) represents the density of the mature population. *α*, *γ*, *τ*, and *β* are all positive constants. *α* is the birth rate, and *γ* is the natural death rate; *τ* is the time from birth to maturity; *β* is the death rate of the mature because of the competition with each other.

And then, many infectious diseases with sage structure have been built and investigated [9–14]. Xiao and Chen [15] improved (1) by separating the population into mature and immature and supposing that only the immature were susceptible to the infection.

Based on the model in [15], supposing that only the mature were susceptible, Jia and Li [16] built a new one as follows:

(2) $$\begin{array}{c} \left\{\begin{array}{c} \dot{x}\left(t\right)=\alpha e^{-\gamma \tau }x\left(t-\tau \right)-\gamma x\left(t\right)-\beta x^{2}\left(t\right)-mx\left(t\right)y\left(t\right)\\ \dot{y}\left(t\right)=mx\left(t\right)y\left(t\right)-\gamma y\left(t\right)-cy\left(t\right)-gy\left(t\right)\\ \dot{z}\left(t\right)=\alpha x\left(t\right)-\gamma z\left(t\right)-\alpha e^{-\gamma \tau }x\left(t-\tau \right)\\ \dot{R}\left(t\right)=gy\left(t\right)-\gamma R\left(t\right) \end{array}\right., \end{array}$$

where *x*(*t*), *y*(*t*), and *R*(*t*) are the susceptible, infectious, and recovered mature population densities, respectively; *z*(*t*) denotes the immature population density. All the parameters are positive constants. *α*, *β*, *γ*, and *τ* are the same as those in (1); *m* is the transmission coefficient describing the infection between the susceptible and the infectious; *c* is the death rate because of the epidemic; *g* is the recovery rate; *αe*^−*γτ*^*x*(*t* − *τ*) denotes the population who were born at *t* − *τ* and survive at *t*.

The article "Stability and Hopf Bifurcation Analysis of an Epidemic Model with Time Delay" was retracted in 2023. Reasons: signs of a paper mill; suspected computer-generated content; unreliable results or conclusions; concerns about the data.

In systems (1) and (2), the time delay was also taken into consideration. Indeed, time delay plays an important role in the epidemic system, making the models more accurate. In recent years, delays have been introduced in more and more epidemic and predator-prey systems [17–19].

In this paper, on the basis of (2), we further assume that

1. Both the susceptible and the infectious have fertility, while in (2), only the susceptible is fertile
2. For the infectious, there is competition with all the susceptible and the infectious, while for the susceptible, there is only competition between generations

Meanwhile, all the death of the susceptible, the same as that in (1), is only due to the competition. To simplify model (2), we denote *γ* + *c* + *g* = *d*, and let *b*(*x*(*t*) + *y*(*t*)) present the transmission from immature to mature.

As a consequence, the new epidemic model could be described as follows:

(3) $$\begin{array}{c} \left\{\begin{array}{c} \dot{x}\left(t\right)=b\left(x\left(t\right)+y\left(t\right)\right)-w\left(x\left(t-\tau \right)+y\left(t-\tau \right)\right)x\left(t\right)-mx\left(t\right)y\left(t\right)\\ \dot{y}\left(t\right)=mx\left(t\right)y\left(t\right)-w\left(x\left(t\right)+y\left(t\right)\right)y\left(t\right)-dy\left(t\right)\\ \dot{z}\left(t\right)=\alpha \left(x\left(t\right)+y\left(t\right)\right)-\gamma z\left(t\right)-b\left(x\left(t\right)+y\left(t\right)\right)\\ \dot{R}\left(t\right)=gy\left(t\right)-\gamma R\left(t\right) \end{array}\right., \end{array}$$

where *w* is the death rate of the mature because of the competition.

The article "Stability and Hopf Bifurcation Analysis of an Epidemic Model with Time Delay" was retracted in 2023. Reasons: signs of a paper mill; suspected computer-generated content; unreliable results or conclusions; concerns about the data.

We can notice that *z*(*t*) depends on *x*(*t*) and *y*(*t*) and *R*(*t*) depends on *y*(*t*); however, *x*(*t*) and *y*(*t*) have nothing to do with *z*(*t*) and *R*(*t*). According to Qu and Wei [20], we will mainly focus on *x*(*t*) and *y*(*t*), that is,

(4) $$\begin{array}{c} \left\{\begin{array}{c} \dot{x}\left(t\right)=b\left(x\left(t\right)+y\left(t\right)\right)-w\left(x\left(t-\tau \right)+y\left(t-\tau \right)\right)x\left(t\right)-mx\left(t\right)y\left(t\right)\\ \dot{y}\left(t\right)=mx\left(t\right)y\left(t\right)-\text{w}\left(x\left(t\right)+y\left(t\right)\right)y\left(t\right)-dy\left(t\right) \end{array}.\right. \end{array}$$

The rest of the paper is organized as follows. In Section 2, we calculate the steady states of system (4) and prove the existence and uniqueness of the positive equilibrium in particular. And then, the stability of the two nonzero equilibria and the existence of the Hopf bifurcation are investigated in Sections 3 and 4, respectively. In Section 5, the direction and stability of the Hopf bifurcation at the positive equilibrium are studied by using the center manifold theorem and the normal form theory [21]. And in the last section, some numerical simulations are carried out to validate the theoretical analysis.

## 2. The Existence and Uniqueness of the Positive Equilibrium of the Model

In this section, we discuss the existence of the equilibria of (4) and the positive one in particular.

The equilibria are the solutions of the equations (5),

(5) $$\begin{array}{c} \left\{\begin{array}{c} b\left(x+y\right)-w\left(x+y\right)x-mxy=0\\ \left[mx-w\left(x+y\right)-d\right]y=0 \end{array}\right.. \end{array}$$

Clearly, *E*_1_(0, 0) and *E*_2_(*b*/*w*, 0) are two equilibria of (4).

In the following, we will focus on the existence of the positive equilibrium.

**Theorem 1 .**

If *b*(*m* − *w*) > *dw*, (4) has one positive equilibrium *E*_3_(*x*^∗^, *y*^∗^), where

(6) $$\begin{array}{c} x^{*}=\left(B+\sqrt{∆}\right)\left(2m^{2}\right),y^{*}=\left(m-w\right)\left(B+\sqrt{∆}\right)/\left(2m^{2}w\right)-d/w. \end{array}$$

**Proof**

Positive equilibrium is the positive solution of the equations (7),

(7) $$\begin{array}{c} \left\{\begin{array}{c} b\left(x+y\right)-w\left(x+y\right)x-mxy=0\\ mx-w\left(x+y\right)-d=0 \end{array}\right.. \end{array}$$

From the second equation of (7), we have

(8) $$\begin{array}{c} wy=\left(m-w\right)x-d. \end{array}$$

Taking (8) into the first equation of (7), we can obtain

(9) $$\begin{array}{c} m^{2}x^{2}-\left(bm+dm+dw\right)x+bd=0, \end{array}$$

which leads to

(10) $$\begin{array}{c} ∆=B^{2}-4m^{2}bd={\left(bm+dw-dm\right)}^{2}+4d^{2}mw>0, \end{array}$$

where

(11) $$\begin{array}{c} B=bm+dm+dw. \end{array}$$

Together with

(12) $$\begin{array}{c} x_{1}+x_{2}=\left(bm+dm+dw\right)/m^{2}>0,\text{and }x_{1}x_{2}=bd/m^{2}>0, \end{array}$$

we can know that both of the two solutions of (9) are positive,

where

(13) $$\begin{array}{c} x_{1}=\frac{B-\sqrt{∆}}{2m^{2}}>0\text{and}x_{2}=\frac{B+\sqrt{∆}}{2m^{2}}>0. \end{array}$$

If $x=B-\sqrt{∆}/2m^{2}$,

then,

(14) $$\begin{array}{c} wy=\left(m-w\right)x-d=\left(m-w\right)\frac{\left(B-\sqrt{∆}\right)}{2m^{2}}-d<\left(m-w\right)\frac{B-\left|bm+dw-dm\right|}{2m^{2}}-d\leq \left(m-w\right)\frac{B-\left(bm+dw-dm\right)}{2m^{2}}-d=-\frac{dw}{m}<0. \end{array}$$

So, $x=B-\sqrt{∆}/2m^{2}$ is dropped.

The article "Stability and Hopf Bifurcation Analysis of an Epidemic Model with Time Delay" was retracted in 2023. Reasons: signs of a paper mill; suspected computer-generated content; unreliable results or conclusions; concerns about the data.

If $x=B+\sqrt{∆}/2m^{2}$,

then,

(15) $$\begin{array}{c} wy=\left(m-w\right)\frac{B+\sqrt{∆}}{2m^{2}}-d=\left(m-w\right)\frac{4m^{2}bd}{2m^{2}\left(B-\sqrt{∆}\right)}-d=d\left[\frac{2b\left(m-w\right)}{B-\sqrt{∆}}-1\right]=d\left(B-\sqrt{∆}\right)\left[2b\left(m-w\right)-\left(B-\sqrt{∆}\right)\right]. \end{array}$$

*w* > 0, *d* > 0, and $B-\sqrt{∆}=\sqrt{∆+4m^{2}bd}-\sqrt{∆}>0$, so $y>0⟺2b\left(m-w\right)-\left(B-\sqrt{∆}\right)>0$,

(16) $$\begin{array}{c} ⟺∆>B^{2}-4b\left(m-w\right)B+4b^{2}{\left(m-w\right)}^{2}⟺m^{2}d-\left(m-w\right)\left(bm-bw-bm-dm-dw\right)<0⟺b\left(m-w\right)>dw∴b\left(m-w\right)>dw⟺y>0. \end{array}$$

Then, taking $x=B+\sqrt{∆}/2m^{2}≜x^{*}$ into (8), we have

(17) $$\begin{array}{c} y=\frac{\left(m-w\right)\left(B+\sqrt{∆}\right)}{\left(2m^{2}w\right)}-\frac{d}{w}≜y^{*}. \end{array}$$

Therefore, if *b*(*m* − *w*) > *dw*, (4) has the unique positive equilibrium *E*_3_(*x*^∗^, *y*^∗^).☐

## 3. Stability Analysis of the Equilibrium E_2_(b/w, 0)

In this section, we analyze the stability of the equilibrium *E*_2_(*b*/*w*,  0).

For convenience, the new variables *u*(*t*) = *x*(*t*) − *b*/*w* and *v*(*t*) = *y*(*t*) are introduced, and then, around *E*_2_(*b*/*w*,  0), the system (4) could be linearized as (18):

(18) $$\begin{array}{c} \left\{\begin{array}{c} \dot{u}\left(t\right)=-bu\left(t-\tau \right)-bv\left(t-\tau \right)+bv\left(t\right)-\frac{bm}{w}v\left(t\right)\\ \dot{v}\left(t\right)=\frac{bm}{w}v\left(t\right)-dv\left(t\right)-b\text{v}\left(t\right) \end{array}\right., \end{array}$$

whose characteristic equation is given by

(19) $$\begin{array}{c} \left(\lambda +be^{-\lambda \tau }\right)\left(\lambda +b+d-\frac{bm}{w}\right)=0, \end{array}$$

from which, we can get that

(20) $$\begin{array}{c} \lambda =-\left(b+d-\frac{bm}{w}\right), \end{array}$$

or

(21) $$\begin{array}{c} \lambda +be^{-\lambda \tau }=0. \end{array}$$

Obviously, if *b*(*m* − *w*) > *dw*,

then

(22) $$\begin{array}{c} \lambda =-\left(b+d-\frac{bm}{w}\right)>0, \end{array}$$

which implies that the equilibrium *E*_2_ is unstable.

The article "Stability and Hopf Bifurcation Analysis of an Epidemic Model with Time Delay" was retracted in 2023. Reasons: signs of a paper mill; suspected computer-generated content; unreliable results or conclusions; concerns about the data.

If *b*(*m* − *w*) < *dw*,

then

(23) $$\begin{array}{c} \lambda =-\left(b+d-bm/w\right)<0. \end{array}$$

As a consequence, we will discuss the other roots of (19), that is, the roots of (21), under the condition *b*(*m* − *w*) < *dw*.

For *τ* = 0, equation (21) becomes

(24) $$\begin{array}{c} \lambda +b=0, \end{array}$$

whose root is

(25) $$\begin{array}{c} \lambda =-b<0. \end{array}$$

For *τ* > 0, if *iω*(*ω* > 0) is a root of (21), then

(26) $$\begin{array}{c} i\omega +b\cos\omega \tau -ib\sin\omega \tau =0. \end{array}$$

(27) can be obtained by separating the real and the imaginary parts,

(27) $$\begin{array}{c} \left\{\begin{array}{c} b\cos\omega \tau =0\\ b\sin\omega \tau =\omega \end{array}\right., \end{array}$$

which leads to

(28) $$\begin{array}{c} \omega^{2}=b^{2}, \end{array}$$

from which, we can get the unique positive root

(29) $$\begin{array}{c} \omega_{0}=b. \end{array}$$

Let

(30) $$\begin{array}{c} \tau_{j}=\frac{\pi \left(4j+1\right)}{2\omega_{0}}\;j=0,1,2,\cdots . \end{array}$$

Then, when *τ* = *τ*_*j*_, (21) has a pair of purely imaginary roots ±*iω*_0_.

Suppose

(31) $$\begin{array}{c} \lambda \left(\tau \right)=\alpha \left(\tau \right)+i\omega \left(\tau \right), \end{array}$$

which is the root of (21) such that

(32) $$\begin{array}{c} \alpha \left(\tau_{j}\right)=0,\text{and}\omega \left(\tau_{j}\right)=\omega_{0}. \end{array}$$

To investigate the distribution of *λ*(*τ*), we will discuss the trend of *λ*(*τ*) at *τ* = *τ*_*j*_.

Substituting *λ*(*τ*) into (21) and taking the derivative with respect to *τ*, we can get

(33) $$\begin{array}{c} \frac{d\lambda }{d\tau }-\text{b}e^{-\lambda \tau }\left(\lambda +\tau \frac{d\lambda }{d\tau }\right)=0, \end{array}$$

which yields,

(34) $$\begin{array}{c} {\left[\frac{d\lambda }{d\tau }\right]}^{-1}=\frac{e^{\lambda \tau }}{b\lambda }-\frac{\tau }{\lambda }. \end{array}$$

Together with (27), we have

(35)  signRedλdττ=τj−1=signReeλτbλτ=τj=signRecosω0τ+isinω0τibω0=signsinω0τbω0=signbsinω0τb2ω0=signω0b2ω0=sign1b2>0,

which means that when undergoes *τ* = *τ*_*j*_, *λ*(*τ*) will add a pair of roots with positive real parts. That is, with the increase of *τ*, the number of roots with positive real part is increasing, leading to the change of the stability of the system (4).

Therefore, the distribution of the roots of (21) could be obtained.

**Lemma 1 .**

Let *ω*_0_ and  *τ*_*j*_ ( *j* = 0, 1, 2,  ⋯) be defined by (29) and (30), respectively.

1. If *b*(*m* − *w*) > *dw*, then (19) has at least one positive root
2. If *b*(*m* − *w*) < *dw*, and *τ* = 0, then both roots of (19) are negative
3. If *b*(*m* − *w*) < *dw*, and *τ* > 0, then (19) has a pair of simple imaginary roots ±*iω*_0_ at *τ* = *τ*_*j*_; furthermore, if *τ* < *τ*_0_, then all the roots of (19) have negative real parts; if *τ* ∈ (*τ*_*j*_, *τ*_*j*+1_), (19) has 2(j + 1) roots with positive real parts

Together with condition (35), the Hopf bifurcation theorem [21], and Lemma 2, the following theorem could be stated.

The article "Stability and Hopf Bifurcation Analysis of an Epidemic Model with Time Delay" was retracted in 2023. Reasons: signs of a paper mill; suspected computer-generated content; unreliable results or conclusions; concerns about the data.

**Theorem 2 .**

Let  *τ*_*j*_ (*j* = 0, 1, 2,  ⋯) be defined by (30), then we have

1. If *b*(*m* − *w*) > *dw*, then the equilibrium *E*_2_(*b*/*w*, 0) of (4) is unstable
2. If *b*(*m* − *w*) < *dw*, then the equilibrium *E*_2_(*b*/*w*, 0) is asymptotically stable when *τ* ∈ [0, *τ*_0_), and it is unstable when *τ* > *τ*_0_
3. If *b*(*m* − *w*) < *dw*, then system (4) undergoes a Hopf bifurcation at the equilibrium *E*_2_(*b*/*w*, 0) for *τ* = *τ*_*j*_

## 4. Stability Analysis of Positive Equilibrium *E*_3_(*x*^∗^, *y*^∗^)

In this section, we analyze the stability of the positive equilibrium *E*_3_(*x*^∗^, *y*^∗^).

For convenience, the new variables *u*(*t*) = *x*(*t*) − *x*^∗^ and *v*(*t*) = *y*(*t*) − *y*^∗^ are introduced, and then, around *E*_3_(*x*^∗^, *y*^∗^), the system (4) could be linearized as (36):

(36) $$\begin{array}{c} \left\{\begin{array}{c} \dot{u}\left(t\right)=\left(b+d-mx^{*}-my^{*}\right)u\left(t\right)-wx^{*}u\left(t-\tau \right)+\left(b-mx^{*}\right)v\left(t\right)-wx^{*}v\left(t-\tau \right)\\ \dot{v}\left(t\right)=\left(m-w\right)y^{*}u\left(t\right)-wy^{*}v\left(t\right) \end{array}\right., \end{array}$$

whose characteristic equation is given by

(37) $$\begin{array}{c} \lambda^{2}+\left(wy^{*}-k\right)\lambda +\left(\lambda +my^{*}\right)se^{-\lambda \tau }-kwy^{*}-\left(m-w\right)y^{*}n=0, \end{array}$$

where

(38) $$\begin{array}{c} k=b+d-mx^{*}-my^{*},n=b-mx^{*},\text{s}=wx^{*}. \end{array}$$

For *τ* = 0, equation (37) becomes

(39) $$\begin{array}{c} \lambda^{2}+\left(wy^{*}-k+s\right)\lambda +msy^{*}-kwy^{*}-\left(m-w\right)y^{*}n=0. \end{array}$$

Firstly, computing *λ*_1_*λ*_2_, we have

(40) $$\begin{array}{c} \;\lambda_{1}\lambda_{2}=msy^{*}-kwy^{*}-\left(m-w\right)y^{*}n=y^{*}\left[mwx^{*}-\left(b+d\right)w+m\left(x^{*}+y^{*}\right)w-\left(m-w\right)b+\left(m-w\right)mx^{*}\right]=y^{*}\left[m^{2}x^{*}+mwx^{*}+m\left(mx^{*}-wx^{*}-d\right)-\left(dw+bm\right)\right]=y^{*}\sqrt{\Delta }, \end{array}$$

where Δ is the same as that in (10).

So,

(41) $$\begin{array}{c} \lambda_{1}\lambda_{2}=msy^{*}-kwy^{*}-\left(m-w\right)y^{*}n>0, \end{array}$$

which implies that the real parts of  *λ*_1_ and *λ*_2_ have the same signs.

Then, (*λ*_1_ + *λ*_2_) is calculated:

(42) $$\begin{array}{c} \lambda_{1}+\lambda_{2}=-\left(wy^{*}-k+s\right)=\left(b+d\right)-m\left(x^{*}+y^{*}\right)y^{*}=b+mx^{*}-w\left(x^{*}+y^{*}\right)-mx^{*}-w\left(x^{*}+y^{*}\right)-my^{*}=-\frac{m{y^{*}}^{2}}{x^{*}+y^{*}}-w\left(x^{*}+y^{*}\right)<0. \end{array}$$

Together with (41), we can get that both the real parts of the two roots of (39) are negative.

The article "Stability and Hopf Bifurcation Analysis of an Epidemic Model with Time Delay" was retracted in 2023. Reasons: signs of a paper mill; suspected computer-generated content; unreliable results or conclusions; concerns about the data.

For *τ* > 0, equation (37) can be rewritten as

(43) $$\begin{array}{c} \lambda^{2}+r\lambda +\left(s\lambda +c\right)e^{-\lambda \tau }+p=0, \end{array}$$

where

(44) $$\begin{array}{c} r=\left(wy^{*}-k\right),s=wx^{*},c=msy^{*},p=-kwy^{*}-\left(m-w\right)y^{*}n. \end{array}$$

If *iω*(*ω* > 0) is a root of (37), then

(45) $$\begin{array}{c} -\omega^{2}+ir\omega +is\omega \cos\omega \tau +sw\sin\omega \tau +c\cos\omega \tau -ic\sin\omega \tau +p=0. \end{array}$$

Separating the real and the imaginary parts, we have

(46) $$\begin{array}{c} \left\{\begin{array}{c} c\cos\omega \tau +s\omega \sin\omega \tau =\omega^{2}-p\\ c\sin\omega \tau -s\omega \cos\omega \tau =r\omega \end{array},\right. \end{array}$$

which leads to

(47) $$\begin{array}{c} \omega^{4}-\left(2p-r^{2}+s^{2}\right)\omega^{2}+p^{2}-c^{2}=0. \end{array}$$

Let *z* = *ω*^2^ > 0, and then, (47) can be rewritten as

(48) $$\begin{array}{c} z^{2}-\left(2p-r^{2}+s^{2}\right)z+p^{2}-c^{2}=0. \end{array}$$

Firstly, computing *z*_1_*z*_2_, we get

(49) $$\begin{array}{c} z_{1}z_{2}=p^{2}-c^{2}=\left(p+c\right)\left(p-c\right), \end{array}$$

where

(50) $$\begin{array}{c} p-c=msy^{*}-kwy^{*}-\left(m-w\right)y^{*}n>0, \end{array}$$

has been proved in (41).

Then, we will calculate

(51) $$\begin{array}{c} p+c=-msy^{*}-kwy^{*}-\left(m-w\right)y^{*}n=y^{*}\left[-mwx^{*}-\left(b+d\right)w+m\left(x^{*}+y^{*}\right)w-\left(m-w\right)b+\left(m-w\right)mx^{*}\right]=y^{*}\left[m^{2}x^{*}-mwx^{*}+mwy^{*}-\left(dw+bm\right)\right]=y^{*}\left[\frac{m-w}{m}\left(\text{B}+\sqrt{\Delta }\right)-B\right]=\frac{y^{*}}{m}\left[\left(m-w\right)\sqrt{\Delta }-wB\right]. \end{array}$$

If H(4-1): $\left(m-w\right)\sqrt{\Delta }-wB<0$,

then

(52) $$\begin{array}{c} p+c<0, \end{array}$$

and then,

(53) $$\begin{array}{c} z_{1}z_{2}<0, \end{array}$$

which implies that (48) has one unique positive solution *z*_0_ = *ω*_0_^2^,

where

(54) $$\begin{array}{c} \omega_{0}={\left\{\frac{2p-r^{2}+s^{2}+\sqrt{{\left(2p-r^{2}+s^{2}\right)}^{2}-4\left(p^{2}-c^{2}\right)}}{2}\right\}}^{1/2}. \end{array}$$

If H(4-2): $\left(m-w\right)\sqrt{\Delta }-wB>0$,

then

(55) $$\begin{array}{c} p+c>0, \end{array}$$

and then,

(56) $$\begin{array}{c} z_{1}z_{2}>0, \end{array}$$

Let

(57) $$\begin{array}{c} {∆}_{1}={\left(2p-r^{2}+s^{2}\right)}^{2}-4\left(p^{2}-c^{2}\right). \end{array}$$

If ∆_1_ < 0, then (48) has no real roots.

The article "Stability and Hopf Bifurcation Analysis of an Epidemic Model with Time Delay" was retracted in 2023. Reasons: signs of a paper mill; suspected computer-generated content; unreliable results or conclusions; concerns about the data.

If ∆_1_ > 0 and *z*_1_ + *z*_2_ = 2*p* − *r*^2^ + *s*^2^ < 0, then (48) has two negative roots, and there no positive *ω* for (47);

If ∆_1_ > 0 and *z*_1_ + *z*_2_ = 2*p* − *r*^2^ + *s*^2^ > 0,

then (48) has two positive roots, and there are two positive *ω* for (47), which are

(58) $$\begin{array}{c} \omega_{\pm }={\left\{\frac{2p-r^{2}+s^{2}\pm \sqrt{{\left(2p-r^{2}+s^{2}\right)}^{2}-4\left(p^{2}-c^{2}\right)}}{2}\right\}}^{1/2}. \end{array}$$

**Lemma 2 .**

1. If $\left(m-w\right)\sqrt{\Delta }-wB<0$, then (47) has one positive root *ω*_0_
2. When $\left(m-w\right)\sqrt{\Delta }-wB>0$, if ∆_1_ < 0, or *z*_1_ + *z*_2_ = 2*p* − *r*^2^ + *s*^2^ < 0, then (47) has no positive roots
3. When $\left(m-w\right)\sqrt{\Delta }-wB>0$, if ∆_1_ > 0 and *z*_1_ + *z*_2_ = 2*p* − *r*^2^ + *s*^2^ > 0, then (47) has two positive roots

In the following, we will discuss the expression of *τ*_*j*_.

**Lemma 3 .**

If

(59) $$\begin{array}{c} \left\{\begin{array}{c} \cos\left(at\right)=f\left(a\right)\\ \sin\left(at\right)=g\left(a\right) \end{array}\right., \end{array}$$

where *a* > 0, *t* > 0, then

1. If *f*(*a*) > 0, *g*(*a*) > 0, then

(60) $$\begin{array}{c} at=\arccos\left(f\left(a\right)\right)+2j\pi ,\text{or }at=\arcsin\left(g\left(a\right)\right)+2j\pi \end{array}$$

(2) If *f*(*a*) < 0, *g*(*a*) > 0, then

(61) $$\begin{array}{c} at=\arccos\left(f\left(a\right)\right)+2j\pi ,\text{or }at=\pi -\arcsin\left(g\left(a\right)\right)+2j\pi \end{array}$$

(3) If *f*(*a*) > 0, *g*(*a*) < 0, then

(62) $$\begin{array}{c} at=2\pi -\arccos\left(f\left(a\right)\right)+2j\pi ,\text{or }at=2\pi +\arcsin\left(g\left(a\right)\right)+2j\pi \end{array}$$

(4) If *f*(*a*) < 0, *g*(*a*) < 0, then

(63) $$\begin{array}{c} at=2\pi -\arccos\left(f\left(a\right)\right)+2j\pi ,\text{or }at=\pi -\arcsin\left(g\left(a\right)\right)+2j\pi \end{array}$$

In conclusion,

1. If *g*(*a*) > 0, then *at* = arccos(*f*(*a*)) + 2*jπ*
2. If *g*(*a*) < 0, then *at* = 2*π* − arccos(*f*(*a*)) + 2*jπ*,

where *j* = 0, 1, 2, ⋯

According to (46), we have

(64) $$\begin{array}{c} \left\{\begin{array}{c} \cos\omega \tau =\frac{c\left(\omega^{2}-p\right)-sr\omega^{2}}{c^{2}+s^{2}\omega^{2}}=f\left(\omega \right)\\ \sin\omega \tau =\frac{s\omega \left(\omega^{2}-p\right)+cr\omega }{c^{2}+s^{2}\omega^{2}}=g\left(\omega \right) \end{array}.\right. \end{array}$$

If $\left(m-w\right)\sqrt{\Delta }-wB<0$, substituting *ω*_0_ defined in (54) into (64), we can get *f*(*ω*_0_) and *g*(*ω*_0_). Together with Lemma 5, the expression of *τ*_*j*_ could be obtained.

If

(65) $$\begin{array}{c} g\left(\omega_{0}\right)>0, \end{array}$$

then

(66) $$\begin{array}{c} \tau_{j}=\frac{1}{\omega_{0}}\left\{\arccos\left[\frac{c\left(\omega_{0}^{2}-p\right)-sr\omega_{0}^{2}}{c^{2}+s^{2}\omega_{0}^{2}}\right]+2\pi j\right\},\;j=0,1,2,\cdots . \end{array}$$

If

(67) $$\begin{array}{c} g\left(\omega_{0}\right)<0, \end{array}$$

then

(68) $$\begin{array}{c} \tau_{j}=\frac{1}{\omega_{0}}\left\{2\pi -\arccos\left[\frac{c\left(\omega_{0}^{2}-p\right)-sr\omega_{0}^{2}}{c^{2}+s^{2}\omega_{0}^{2}}\right]+2\pi j\right\},\;j=0,1,2,\cdots . \end{array}$$

That is, when *τ* = *τ*_*j*_, the characteristic equation (37) has a pair of purely imaginary roots ±*iω*_0_.

The article "Stability and Hopf Bifurcation Analysis of an Epidemic Model with Time Delay" was retracted in 2023. Reasons: signs of a paper mill; suspected computer-generated content; unreliable results or conclusions; concerns about the data.

Suppose *λ*(*τ*) = *α*(*τ*) + *iω*(*τ*) is the root of (37), and then, we have

(69) $$\begin{array}{c} \alpha \left(\tau_{j}\right)=0,\text{and}\omega \left(\tau_{j}\right)=\omega_{0}. \end{array}$$

To investigate the distribution of the *λ*(*τ*), we will discuss the trend of *λ*(*τ*) at *τ* = *τ*_*j*_.

Substituting *λ*(*τ*) into (37) and taking the derivative with respect to *τ*, we can get

(70) $$\begin{array}{c} \left[2\lambda +r+se^{-\lambda \tau }-e^{-\lambda \tau }\left(s\lambda +c\right)\tau \right]\frac{d\lambda }{d\tau }=\lambda e^{-\lambda \tau }\left(s\lambda +c\right), \end{array}$$

which leads to

(71) $$\begin{array}{c} {\left[\frac{d\lambda }{d\tau }\right]}^{-1}=\frac{e^{\lambda \tau }\left(s\lambda +c\right)+s}{\lambda \left(s\lambda +c\right)}-\frac{\tau }{\lambda }. \end{array}$$

Together with (46) and (54), we have

(72) signRedλdττ=τj−1=signReeλτsλ+c+sλsλ+cτ=τj=signRecosω0τ+isinω0τ2iω0+r+siω0isω0+c=signc2ω0cosω0τ+rsinω0τ−sω0rcosω0τ−2ω0sinω0τ+s=sign2ω0ω02−p+rrω0=sign2p−r2+s2+2p−r2+s22−4p2−c2−2p−r2+s2=sign2p−r2+s22−4p2−c2>0,

which means that when undergoes *τ* = *τ*_*j*_, *λ*(*τ*) will add a pair of roots with positive real parts. That is, with the increase of *τ*, the number of roots with positive real part is increasing, leading to the change of the stability of the system (4).

If $\left(m-w\right)\sqrt{\Delta }-wB>0$, ∆_1_ > 0 and *z*_1_ + *z*_2_ = 2*p* − *r*^2^ + *s*^2^ > 0, then *f*(*ω*_0_) and *g*(*ω*_0_) could be calculated by substituting *ω*_±_ defined in (58) into (64). According to Lemma 5, we can get the expression of *τ*_*j*_^±^:

If

(73) $$\begin{array}{c} g\left(\omega_{\pm }\right)>0, \end{array}$$

then

(74) $$\begin{array}{c} \tau_{j}^{\pm }=\frac{1}{\omega_{\pm }}\left\{\arccos\left[\frac{c\left(\omega_{\pm }^{2}-p\right)-sr\omega_{\pm }^{2}}{c^{2}+s^{2}\omega_{\pm }^{2}}\right]+2\pi j\right\},\;j=0,1,2,\cdots . \end{array}$$

If

(75) $$\begin{array}{c} g\left(\omega_{\pm }\right)<0, \end{array}$$

then

(76) $$\begin{array}{c} \tau_{j}^{\pm }=\frac{1}{\omega_{\pm }}\left\{2\pi \left(j+1\right)-\arccos\left[\frac{c\left(\omega_{\pm }^{2}-p\right)-sr\omega_{\pm }^{2}}{c^{2}+s^{2}\omega_{\pm }^{2}}\right]\right\},\;j=0,1,2,\cdots . \end{array}$$

That is, when *τ* = *τ*_*j*_^±^, the characteristic equation (37) has a pair of purely imaginary roots ±*iω*_±_.

The article "Stability and Hopf Bifurcation Analysis of an Epidemic Model with Time Delay" was retracted in 2023. Reasons: signs of a paper mill; suspected computer-generated content; unreliable results or conclusions; concerns about the data.

Let *λ*(*τ*) = *α*(*τ*) + *iω*(*τ*) be the root of (37), satisfying

(77) $$\begin{array}{c} \alpha \left(\tau_{j}^{\pm }\right)=0,\text{and}\omega \left(\tau_{j}^{\pm }\right)=\omega_{\pm }. \end{array}$$

To investigate the distribution of the *λ*(*τ*), we will discuss the trend of *λ*(*τ*) at *τ* = *τ*_*j*_^±^.

Using the same method, we have

(78) signRedλdττ=τj±−1=sign2ω±2−2p−r2+s2=sign2p−r2+s2±2p−r2+s22−4p2−c2−2p−r2+s2=sign±2p−r2+s22−4p2−c2=sign±∆1.

This implies that

(79) $$\begin{array}{c} {\left[\frac{d\lambda }{d\tau }\right]}_{\tau =\tau_{j}^{+}}>0, \end{array}$$

and

(80) $$\begin{array}{c} {\left[\frac{d\lambda }{d\tau }\right]}_{\tau =\tau_{j}^{-}}<0, \end{array}$$

which means that when undergoes *τ* = *τ*_*j*_^+^, *λ*(*τ*) will add a pair of roots with positive real parts, while undergoes *τ* = *τ*_*j*_^−^, *λ*(*τ*) will lose a pair of roots with positive real parts; if *τ*_*j*_^−^ > *τ*_*j*+1_^+^, then the characteristic equation (37) must have roots with positive real parts for *τ* > *τ*_*j*+1_^+^.

In conclusion, the distribution of the roots of (37) could be obtained.

**Lemma 4 .**

Let *ω*_0_ be defined by (54), and  *τ*_*j*_ ( *j* = 0, 1, 2,  ⋯) be defined by (66) or (68), and *ω*_±_ be defined by (58), and *τ*_*j*_^±^ ( *j* = 0, 1, 2,  ⋯) be defined by (74) or (76), respectively.

1. When $\left(m-w\right)\sqrt{\Delta }-wB>0$, if ∆_1_ < 0, or *z*_1_ + *z*_2_ = 2*p* − *r*^2^ + *s*^2^ < 0, then all the roots of (37) are with negative real parts
2. When $\left(m-w\right)\sqrt{\Delta }-wB<0$, (37) has a pair of simple imaginary roots ±*iω*_0_ at *τ* = *τ*_*j*_; furthermore, if *τ* ∈ [0, *τ*_0_), then all the roots of (37) are with negative real parts; if *τ* ∈ (*τ*_*j*_, *τ*_*j*+1_), then (37) has 2(j + 1) roots with positive real parts
3. When $\left(m-w\right)\sqrt{\Delta }-wB>0$, if ∆_1_ > 0, and *z*_1_ + *z*_2_ = 2*p* − *r*^2^ + *s*^2^ > 0, then (37) has a pair of simple imaginary roots ±*iω*_±_ at *τ* = *τ*_*j*_^±^; if *τ* ∈ [0, *τ*_0_^+^) or *τ* ∈ (*τ*_*j*_^−^, *τ*_*j*+1_^+^), then all the roots of (37) are with negative real parts; if *τ* ∈ (*τ*_*j*+1_^+^, *τ*_*j*+1_^−^), then (37) has a pair of roots with positive real parts; if *τ*_*h*_^−^ > *τ*_*h*+1_^+^, for *τ* > *τ*_*h*+1_^+^, (37) must have roots with positive real parts

Together with conditions (72) and (78), the Hopf bifurcation theorem [21], and Lemma 6, the following theorem could be stated.

**Theorem 3 .**

Let  *τ*_*j*_ ( *j* = 0, 1, 2,  ⋯) be defined by (66) or (68), and *τ*_*j*_^±^ ( *j* = 0, 1, 2,  ⋯) be defined by (74) or (76), respectively, and then we have

1. When $\left(m-w\right)\sqrt{\Delta }-wB>0$, if ∆_1_ < 0, or *z*_1_ + *z*_2_ = 2*p* − *r*^2^ + *s*^2^ < 0, the equilibrium *E*_3_(*x*^∗^, *y*^∗^) of (4) is asymptotically stable
2. When $\left(m-w\right)\sqrt{\Delta }-wB<0$, then the equilibrium *E*_3_(*x*^∗^, *y*^∗^) is asymptotically stable when *τ* ∈ [0, *τ*_0_), and it is unstable when *τ* > *τ*_0_. System (4) undergoes a Hopf bifurcation at the equilibrium *E*_3_(*x*^∗^, *y*^∗^) for *τ* = *τ*_*j*_
3. When $\left(m-w\right)\sqrt{\Delta }-wB>0$, if ∆_1_ > 0, and *z*_1_ + *z*_2_ = 2*p* − *r*^2^ + *s*^2^ > 0, then there is a positive *h*, such that when *τ* ∈ [0, *τ*_0_^+^) ∪ (*τ*_0_^−^, *τ*_1_^+^) ∪ (*τ*_1_^−^, *τ*_2_^+^) ∪ ⋯∪(*τ*_*h*−1_^−^, *τ*_*h*_^+^), the equilibrium *E*_3_(*x*^∗^, *y*^∗^) is asymptotically stable, and it is unstable when *τ* ∈ (*τ*_0_^+^, *τ*_0_^−^) ∪ (*τ*_1_^+^, *τ*_1_^−^) ∪ (*τ*_2_^+^, *τ*_2_^−^) ∪ ⋯∪(*τ*_*h*−1_^+^, *τ*_*h*−1_^−^) ∪ (*τ*_*h*_^+^, +∞). We call that system (4) undergoes (*h* + 1) switches

System (4) undergoes a Hopf bifurcation at the equilibrium *E*_3_(*x*^∗^, *y*^∗^) for *τ* = *τ*_*j*_^±^.

The article "Stability and Hopf Bifurcation Analysis of an Epidemic Model with Time Delay" was retracted in 2023. Reasons: signs of a paper mill; suspected computer-generated content; unreliable results or conclusions; concerns about the data.

## 5. The Direction and Stability of Hopf Bifurcation at *E*_3_(*x*^∗^, *y*^∗^)

In the previous section, we have already gotten some conditions making that the system (4) undergoes a Hopf bifurcation at the positive equilibrium *E*_3_(*x*^∗^, *y*^∗^) when *τ* = *τ*_*j*_^±^, *j* = 0, 1, 2,  ⋯. In this section, under the conditions in Theorem 7, the direction of Hopf bifurcation and stability of the periodic solutions from *E*_3_ will be investigated by using the center manifold and normal form theories [21].

Without loss of the generality, let $\bar{\tau }$ be the critical value of *τ* = *τ*_*j*_^+^(*τ*_*j*_^−^), *j* = 0, 1, 2,  ⋯.

For convenience, let $\tau =\bar{\tau }+\rho$, *ρ* ∈ *R*, *u*(*t*) = *x*(*τt*) − *x*^∗^, *v*(*t*) = *y*(*τt*) − *y*^∗^, and then system (4) undergoes Hopf bifurcation at *ρ* = 0; with *τ* normalized by the time scaling *t*⟶*t*/*τ*, (4) could be rewritten as

(81) $$\begin{array}{c} \left\{\begin{array}{c} \dot{u}\left(t\right)=\tau \left[b\left(u\left(t\right)+v\left(t\right)+x^{*}+y^{*}\right)-w\left(u\left(t-1\right)+v\left(t-1\right)+x^{*}+y^{*}\right)\left(u\left(t\right)+x^{*}\right)-m\left(u\left(t\right)+x^{*}\right)\left(v\left(t\right)+y^{*}\right)\right]\\ \dot{v}\left(t\right)=\tau \left[m\left(u\left(t\right)+x^{*}\right)\left(v\left(t\right)+y^{*}\right)-d\left(v\left(t\right)+y^{*}\right)-w\left(u\left(t\right)+x^{*}\right)\left(v\left(t\right)+y^{*}\right)\right] \end{array}\right.. \end{array}$$

Choose the space as *C* = *C*([−1, 0], *R*^2^); for any *Φ* = (*Φ*_1_, *Φ*_2_) ∈ *C*, let

(82) $$\begin{array}{c} L_{\rho }\Phi =\left(\bar{\tau }+\rho \right)\left(\frac{m\Phi_{1}\left(0\right)-s\Phi_{1}\left(-1\right)+n\Phi_{2}\left(0\right)-s\Phi_{2}\left(-1\right)}{\left(m-w\right)y^{*}\Phi_{1}\left(0\right)-wy^{*}\Phi_{2}\left(0\right)}\right), \end{array}$$

and

(83) $$\begin{array}{c} f\left(\bar{\tau },\rho \right)=\left(\bar{\tau }+\rho \right)\left(\begin{array}{c} -w\Phi_{1}\left(0\right)\left[\Phi_{1}\left(-1\right)+\Phi_{2}\left(-1\right)\right]-m\Phi_{1}\left(0\right)\Phi_{2}\left(0\right)\\ \left(m-w\right)\Phi_{1}\left(0\right)\Phi_{2}\left(0\right)-w{\Phi_{2}}^{2}\left(0\right) \end{array}\right), \end{array}$$

where *s* and *n* are the same as those in (37).

The article "Stability and Hopf Bifurcation Analysis of an Epidemic Model with Time Delay" was retracted in 2023. Reasons: signs of a paper mill; suspected computer-generated content; unreliable results or conclusions; concerns about the data.

According to Riesz's representation theorem, there is a 2 × 2 matrix *η*(*θ*, *ρ*) (*θ* ∈ [−1, 0]), whose components are bounded variation functions such that

(84) $$\begin{array}{c} L_{\rho }\Phi =\int_{-1}^{0}d\eta \left(\theta ,\rho \right)\Phi \left(\theta \right)\text{ for }\theta \in C. \end{array}$$

In fact, *η*(*θ*, *ρ*) could be chosen as

(85) $$\begin{array}{c} \eta \left(\theta ,\rho \right)=\left(\bar{\tau }+\rho \right)\left(\begin{array}{cc} m & n\\ m-w & wy^{*} \end{array}\right)\delta \left(\theta \right)+\left(\bar{\tau }+\rho \right)\left(\begin{array}{cc} -s & -s\\ 0 & 0 \end{array}\right)\delta \left(\theta +1\right), \end{array}$$

where

(86) $$\begin{array}{c} \delta \left(\theta \right)=\left\{\begin{array}{cc} 0, & \theta =0\\ 1, & \theta \neq 0 \end{array}\right.. \end{array}$$

For any *Φ* ∈ *C*^1^([−1, 0], *R*^2^), we define

(87) $$\begin{array}{c} A\left(\rho \right)\Phi \left(\theta \right)=\left\{\begin{array}{cc} \frac{d\Phi \left(\theta \right)}{d\theta }, & \theta \in \left[-1,0\right)\\ \int_{-1}^{0}d\eta \left(\sigma ,\rho \right)\Phi \left(\sigma \right), & \theta =0 \end{array}\right., \end{array}$$

and

(88) $$\begin{array}{c} R\left(\rho \right)\Phi =\left\{\begin{array}{cc} 0, & \theta \in \left[-1,0\right)\\ f\left(\rho ,\Phi \right)\text{m}, & \theta =0 \end{array}.\right. \end{array}$$

And then, system (4) could be translated into

(89) $$\begin{array}{c} {\dot{x}}_{t}=A\left(\rho \right)x_{t}+R\left(\rho \right)x_{t}, \end{array}$$

where

(90) $$\begin{array}{c} x_{t}=x\left(t+\rho \right)=\left(\frac{u\left(t+\rho \right)}{v\left(t+\rho \right)}\right). \end{array}$$

For Ψ ∈ *C*^1^([−1, 0], (*R*^2^)^∗^), define

(91) $$\begin{array}{c} A^{*}\Psi \left(s\right)=\left\{\begin{array}{cc} -\frac{d\Psi \left(s\right)}{ds}, & s\in \left[-1,0\right)\\ \int_{-1}^{0}d\eta \left(t,0\right)\Psi \left(-t\right),\; & s=0 \end{array},\right. \end{array}$$

and a bilinear form

(92) $$\begin{array}{c} \langle \Psi \left(s\right),\Phi \left(\theta \right)\rangle =\bar{\Psi }\left(0\right)\Phi \left(0\right)-\int_{-1}^{0}\int_{\xi =0}^{\theta }\bar{\Psi }\left(\xi -\theta \right)d\eta \left(\theta \right)\Psi \left(\xi \right)d\xi , \end{array}$$

where

(93) $$\begin{array}{c} \eta \left(\theta \right)=\eta \left(\theta ,0\right). \end{array}$$

According to (87) and (91), we can get that *A*(0) and *A*^∗^ are adjoint operators.

The article "Stability and Hopf Bifurcation Analysis of an Epidemic Model with Time Delay" was retracted in 2023. Reasons: signs of a paper mill; suspected computer-generated content; unreliable results or conclusions; concerns about the data.

From the analysis in Section 4, we know that $\pm i\omega \bar{\tau }$ are a pair of eigenvalues of *A*(0) and also eigenvalues of *A*^∗^, where *ω* is *ω*_+_ or *ω*_−_ defined in (58).

It is easy to verify that vectors *q*(*θ*) and *q*^∗^(*s*) are the eigenvalues of *A*(0) and *A*^∗^ corresponding to the eigenvalues $i\omega \bar{\tau }$ and $-i\omega \bar{\tau }$, where

(94) $$\begin{array}{c} \text{q}\left(\theta \right)={\left(\frac{i\omega +wy^{*}}{\left(m-w\right)y^{*}},1\right)}^{T}e^{i\omega \bar{\tau }\theta },\\ q^{*}\left(s\right)=\bar{B}\left(1,\frac{-i\omega -m+se^{i\omega \bar{\tau }}}{\left(m-w\right)y^{*}}\right)e^{i\omega \bar{\tau }s}. \end{array}$$

For convenience, let

(95) $$\begin{array}{c} \bar{M}=\frac{-i\omega -m+se^{i\omega \bar{\tau }}}{\left(m-w\right)y^{*}},\\ N=\frac{i\omega +wy^{*}}{\left(m-w\right)y^{*}}, \end{array}$$

then

(96) $$\begin{array}{c} \langle q^{*}\left(s\right),q\left(\theta \right)\rangle =B\left\{\left(1,M\right)\left(\frac{N}{1}\right)-\int_{-1}^{0}\int_{\varepsilon =0}^{\theta }\left(1,M\right)e^{-i\omega \bar{\tau }\left(\varepsilon -\theta \right)}d\;\eta \left(\theta \right)\left(\frac{N}{1}\right)e^{i\omega \bar{\tau }\varepsilon }d\varepsilon \right\}=B\left(M+N\right)-B\int_{-1}^{0}\left(1,M\right)\theta e^{i\omega \bar{\tau }\theta }d\;\eta \left(\theta \right)\left(\frac{N}{1}\right)=B\left(M+N\right)-B\left(1,M\right)\int_{-1}^{0}\;d\eta \left(\theta \right)\left(\frac{\theta Ne^{i\omega \bar{\tau }\theta }}{\theta e^{i\omega \bar{\tau }\theta }}\right)=B\left(M+N\right)-B\left(1,M\right)\bar{\tau }\left(\frac{s\left(N+1\right)e^{-i\omega \bar{\tau }}}{0}\right)=B\left(M+N\right)-B\bar{\tau }s\left(N+1\right)e^{-i\omega \bar{\tau }}. \end{array}$$

We choose

(97) $$\begin{array}{c} B={\left[M+N-\bar{\tau }s\left(N+1\right)e^{-i\omega \bar{\tau }}\right]}^{-1}, \end{array}$$

and then,

(98) $$\begin{array}{c} \begin{array}{cc} \langle q^{*}\left(s\right),q\left(\theta \right)\rangle =1, & \langle q\left(\theta \right),q^{*}\left(s\right)\rangle =0 \end{array}. \end{array}$$

Using the same method as that in [21], the center manifold *C*_0_ at *ρ* = 0 is first computed. Suppose that *x*_*t*_ is the solution of (81) when *ρ* = 0, and define

(99) zt=q∗,xtθ,Wt,θ=xtθ−2Reztqθ.

The article "Stability and Hopf Bifurcation Analysis of an Epidemic Model with Time Delay" was retracted in 2023. Reasons: signs of a paper mill; suspected computer-generated content; unreliable results or conclusions; concerns about the data.

Then, on the center manifold *C*_0_, we can get that

(100) $$\begin{array}{c} W\left(t,\theta \right)=W\left(z\left(t\right),\bar{z}\left(t\right),\theta \right), \end{array}$$

where

(101) $$\begin{array}{c} W\left(z\left(t\right),\bar{z}\left(t\right),\theta \right)=W_{20}\left(\theta \right)\frac{z^{2}}{2}+W_{11}\left(\theta \right)z\bar{z}+W_{02}\left(\theta \right)\frac{{\bar{z}}^{2}}{2}+W_{30}\left(\theta \right)\frac{z^{3}}{2}+\cdots . \end{array}$$

In the direction *q*^∗^ and ${\bar{q}}^{*}$, z and $\bar{z}$ are local coordinates for center manifold *C*_0_. It is not difficult to note that when *x*_*t*_ is real, *W* is real. And the real solutions are considered only.

For any solution *x*_*t*_ ∈ *C*_0_, since *ρ* = 0, we can get that

(102) z˙t=q∗,xt˙=iωτ¯zt+q¯∗0f0,Wzt,z¯t,θ+2Reztq0≝iωτ¯zt+q¯∗0f0z,z¯,

where

(103) $$\begin{array}{c} f_{0}\left(z,\bar{z}\right)=f_{z^{2}}\frac{z^{2}}{2}+f_{{\bar{z}}^{2}}\frac{{\bar{z}}^{2}}{2}+f_{z\bar{z}}z\bar{z}+f_{z^{2}\bar{z}}\frac{z^{2}\bar{z}}{2}+\cdots . \end{array}$$

We rewrite

(104) $$\begin{array}{c} \dot{z}\left(t\right)=i\omega \bar{\tau }z\left(t\right)+g\left(z,\bar{z}\right), \end{array}$$

with

(105) $$\begin{array}{c} g\left(z,\bar{z}\right)={\bar{q}}^{*}\left(0\right)f_{0}\left(z,\bar{z}\right)=g_{20}\frac{z^{2}}{2}+g_{11}z\bar{z}+g_{02}\frac{{\bar{z}}^{2}}{2}+g_{21}\frac{z^{2}\bar{z}}{2}+\cdots . \end{array}$$

Together with (83), we have

(106) $$\begin{array}{c} g\left(z,\bar{z}\right)={\bar{q}}^{*}\left(0\right)f\left(0,W\left(z\left(t\right),\bar{z}\left(t\right),\theta \right)\right)={\bar{q}}^{*}\left(0\right)f\left(0,x_{t}\right)=\left(1,M\right)B\bar{\tau }\left(\begin{array}{c} -w\left(W^{1}\left(0\right)+zN+\bar{z}\bar{N}\right)\left[W^{1}\left(-1\right)+zNe^{-i\omega \bar{\tau }}+\bar{z}\bar{N}e^{i\omega \bar{\tau }}+\left(W^{2}\left(-1\right)+ze^{-i\omega \bar{\tau }}+\bar{z}e^{i\omega \bar{\tau }}\right)\right]-m\left(W^{1}\left(0\right)+zN+\bar{z}\bar{N}\right)\left(W^{2}\left(0\right)+z+\bar{z}\right)\\ \cdots \cdots \cdots \cdots \cdots \cdots \cdots \cdots \cdots \cdots \cdots \cdots \cdots \cdots \cdots \cdots \cdots \cdots \cdots \cdots \cdots \cdots \cdots \cdots \cdots \cdots \cdots \cdots \\ \left(m-w\right)\left(W^{1}\left(0\right)+zN+\bar{z}\bar{N}\right)\left(W^{2}\left(0\right)+z+\bar{z}\right)-w{\left(W^{2}\left(0\right)+z+\bar{z}\right)}^{2} \end{array}\right)=-2B\bar{\tau }\left[w\left(N^{2}e^{-i\omega \bar{\tau }}+Ne^{-i\omega \bar{\tau }}\right)+mN\right]\frac{z^{2}}{2}-B\bar{\tau }\left[wN\left(\bar{N}+1\right)e^{i\omega \bar{\tau }}+w\bar{N}\left(N+1\right)e^{-i\omega \bar{\tau }}+m\left(N+\bar{N}\right)\right]z\bar{z}-2B\bar{\tau }\left[w\bar{N}\left(N+1\right)e^{i\omega \bar{\tau }}+m\bar{N}\right]\frac{{\bar{z}}^{2}}{2}-B\bar{\tau }\left\{w\left[W_{20}^{1}\left(0\right)\left(\bar{N}+1\right)e^{i\omega \bar{\tau }}+2W_{11}^{1}\left(0\right)\left(N+1\right)e^{-i\omega \bar{\tau }}+2N\left(W_{11}^{2}\left(-1\right)+W_{11}^{1}\left(-1\right)\right)\right]+m\left[W_{20}^{1}\left(0\right)+2W_{11}^{1}\left(0\right)+2NW_{11}^{2}\left(0\right)+\bar{N}W_{20}^{2}\left(0\right)\right]\right\}\frac{z^{2}\bar{z}}{2}+2B\bar{\tau }M\left[\left(m-w\right)N-w\right]\frac{z^{2}}{2}+B\bar{\tau }M\;\left[\left(N+\bar{N}\right)\left(m-w\right)-2w\right]z\bar{z}+2B\bar{\tau }M\left[\left(m-w\right)\bar{N}-w\right]\frac{{\bar{z}}^{2}}{2}+B\bar{\tau }M\left\{\left(m-w\right)\left[W_{20}^{1}\left(0\right)+2W_{11}^{1}\left(0\right)+2NW_{11}^{2}\left(0\right)\right]-2w\left(2W_{11}^{2}\left(0\right)+W_{20}^{2}\left(0\right)\right)\right\}\;\frac{z^{2}\bar{z}}{2}. \end{array}$$

Comparing with (105), we get

(107) $$\begin{array}{c} g_{20}=-2B\bar{\tau }\left[w\left(N^{2}e^{-i\omega \bar{\tau }}+Ne^{-i\omega \bar{\tau }}\right)+mN\right]+2B\bar{\tau }M\left[\left(m-w\right)N-w\right],\\ g_{11}=-B\bar{\tau }\left[wN\left(\bar{N}+1\right)e^{i\omega \bar{\tau }}+w\bar{N}\left(N+1\right)e^{-i\omega \bar{\tau }}+m\left(N+\bar{N}\right)\right]+B\bar{\tau }M\;\left[\left(N+\bar{N}\right)\left(m-w\right)-2w\right]\\ g_{02}=-2B\bar{\tau }\left[w\bar{N}\left(N+1\right)e^{i\omega \bar{\tau }}+m\bar{N}\right]+2B\bar{\tau }M\left[\left(m-w\right)\bar{N}-w\right]\\ g_{21}=-B\bar{\tau }\left\{w\left[W_{20}^{1}\left(0\right)\left(\bar{N}+1\right)e^{i\omega \bar{\tau }}+2W_{11}^{1}\left(0\right)\left(N+1\right)e^{-i\omega \bar{\tau }}+2N\left(W_{11}^{2}\left(-1\right)+W_{11}^{1}\left(-1\right)\right)\right]+m\left[W_{20}^{1}\left(0\right)+2W_{11}^{1}\left(0\right)+2NW_{11}^{2}\left(0\right)+\bar{N}W_{20}^{2}\left(0\right)\right]\right\}+B\bar{\tau }M\left\{\left(m-w\right)\left[W_{20}^{1}\left(0\right)+2W_{11}^{1}\left(0\right)+2NW_{11}^{2}\left(0\right)\right]-2w\left(2W_{11}^{2}\left(0\right)+W_{20}^{2}\left(0\right)\right)\right\}. \end{array}$$

All the numbers in the expressions of *g*_20_,  *g*_11_, and  *g*_02_ are known; however, *W*_20_ and *W*_11_ in *g*_21_ are unknown, which will be computed in the following.

The article "Stability and Hopf Bifurcation Analysis of an Epidemic Model with Time Delay" was retracted in 2023. Reasons: signs of a paper mill; suspected computer-generated content; unreliable results or conclusions; concerns about the data.

From (89) and (99),

(108) W˙=xt˙−z˙q−z¯˙q¯=AW−2Req¯∗0f0qθ,θ∈−1,0AW−2Req¯∗0f0q0+f0,θ=0≝AW+Hzt,z¯t,θ,

where

(109) $$\begin{array}{c} H\left(z\left(t\right),\bar{z}\left(t\right),\theta \right)=H_{20}\left(\theta \right)\frac{z^{2}}{2}+H_{11}\left(\theta \right)z\bar{z}+H_{02}\left(\theta \right)\frac{{\bar{z}}^{2}}{2}+\cdots . \end{array}$$

When *θ* ∈ [−1, 0],

(110) $$\begin{array}{c} H\left(z\left(t\right),\bar{z}\left(t\right),\theta \right)=-{\bar{q}}^{*}\left(0\right)f_{0}q\left(\theta \right)-q^{*}\left(0\right)\bar{f_{0}}\bar{q}\left(\theta \right)=-g\left(z,\bar{z}\right)q\left(\theta \right)-\bar{g}\left(z,\bar{z}\right)\bar{q}\left(\theta \right). \end{array}$$

Comparing the coefficients in the expansions of (109) and (110), we have

(111) $$\begin{array}{c} \left\{\begin{array}{c} H_{20}\left(\theta \right)=-g_{20}q\left(\theta \right)-{\bar{g}}_{02}\bar{q}\left(\theta \right)\\ H_{11}\left(\theta \right)=-g_{11}q\left(\theta \right)-{\bar{g}}_{11}\bar{q}\left(\theta \right) \end{array}\right.. \end{array}$$

Taking (5-18) into (5-17), we obtain

(112) $$\begin{array}{c} \left(A-2i\omega \bar{\tau }\right)W_{20}\left(\theta \right)=-H_{20}\left(\theta \right)AW_{11}\left(\theta \right)=-H_{11}\left(\theta \right)\cdots . \end{array}$$

By (111) and (112), the following can be gotten

(113) $$\begin{array}{c} {\dot{W}}_{20}\left(\theta \right)=2i\omega \bar{\tau }W_{20}\left(\theta \right)+g_{20}q\left(\theta \right)+{\bar{g}}_{20}\bar{q}\left(\theta \right),\\ {\dot{W}}_{11}\left(\theta \right)=g_{11}q\left(\theta \right)+{\bar{g}}_{11}\bar{q}\left(\theta \right). \end{array}$$

Because

(114) $$\begin{array}{c} q\left(\theta \right)=q\left(0\right)e^{i\omega \bar{\tau }\theta }, \end{array}$$

by integration, we have

(115) $$\begin{array}{c} W_{20}\left(\theta \right)=\frac{ig_{20}}{\omega \bar{\tau }}q\left(0\right)e^{i\omega \bar{\tau }\theta }+\frac{i{\bar{g}}_{20}}{3\omega \bar{\tau }}\bar{q}\left(0\right)e^{-i\omega \bar{\tau }\theta }+E_{1}e^{2i\omega \bar{\tau }\theta }, \end{array}$$

and

(116) $$\begin{array}{c} W_{11}\left(\theta \right)=-\frac{ig_{11}}{\omega \bar{\tau }}q\left(0\right)e^{i\omega \bar{\tau }\theta }+\frac{i{\bar{g}}_{11}}{\omega \bar{\tau }}\bar{q}\left(0\right)e^{-i\omega \bar{\tau }\theta }+E_{2}, \end{array}$$

where *E*_1_ and *E*_2_ are unknown.

From (112) and the definition of A, we obtain

(117) $$\begin{array}{c} \int_{-1}^{0}d\eta \left(\theta \right)W_{20}\left(\theta \right)=2i\omega \bar{\tau }W_{20}\left(\theta \right)-H_{20}\left(\theta \right), \end{array}$$

and

(118) $$\begin{array}{c} \int_{-1}^{0}d\eta \left(\theta \right)W_{11}\left(\theta \right)=-H_{11}\left(\theta \right). \end{array}$$

Then, together with (108), we get

(119) H200=−g20q0−g¯02q¯0+2−wNNe−iωτ¯+1−mNm−wN−wH110=−g11q0−g¯11q¯0+2−wReNNe−iωτ¯+1−mReNm−wReN−w.

Substituting (115) and (119) into (117), we have

(120) $$\begin{array}{c} \left[2i\omega \bar{\tau }I-\int_{-1}^{0}e^{i\omega \bar{\tau }\theta }d\eta \left(\theta \right)\right]E_{1}=2\left(\begin{array}{c} -wN\left[Ne^{-i\omega \bar{\tau }}+1\right]-\left.mN\right)\\ \left(m-w\right)\left.N-w\right) \end{array}\right). \end{array}$$

That is

(121) $$\begin{array}{c} \left(\begin{array}{cc} 2i\omega -m+se^{-2i\omega \bar{\tau }} & -n+se^{-2i\omega \bar{\tau }}\\ -\left(m-w\right)y^{*} & 2i\omega +wy^{*} \end{array}\right)E_{1}=2\left(\begin{array}{c} -wN\left[Ne^{-i\omega \bar{\tau }}+1\right]-\left.mN\right)\\ \left(m-w\right)\left.N-w\right) \end{array}\right), \end{array}$$

from which, *E*_1_ can be determined.

The article "Stability and Hopf Bifurcation Analysis of an Epidemic Model with Time Delay" was retracted in 2023. Reasons: signs of a paper mill; suspected computer-generated content; unreliable results or conclusions; concerns about the data.

By (115), (117), and (119), we have

(122) ∫−10dηθE2=2−wReNNe−iωτ¯+1−mReNm−wReN−w.

That is

(123) −m+s−n+s−m−wy∗wy∗E2=2−wReNNe−iωτ¯+1−mReNm−wReN−w,

from which, *E*_2_ can be determined.

Substituting *E*_1_ and *E*_2_ into (115) and (116), *W*_20_ and *W*_11_ could be obtained; furthermore, *g*_21_ can be calculated.

Then, the important parameters can be obtained:

(124) C10=i2ωτ¯g20g11−2g112−13g022+g212,μ2=−ReC10Reλ′τ¯,β2=2ReC10, T2=−ImC10+μ2Imλ′τ¯ωτ¯,

which determine the quantities of the bifurcation of system (4) at $\tau =\bar{\tau }$, where *μ*_2_ determines the direction of the bifurcation: Hopf bifurcation is subcritical (supercritical) if *μ*_2_ < 0 (*μ*_2_ > 0) and the bifurcating periodic solutions exist for $\tau <\bar{\tau }$ ($\tau >\bar{\tau }$); *β*_2_ determines the stability of the bifurcating periodic solutions, which are stable (unstable) if *β*_2_ < 0 (*β*_2_ > 0); *T*_2_ determines the period of the periodic solutions, which decreases (increases) if *T*_2_ < 0 (*T*_2_ > 0).

From (78) in Section 4, we know that Reλ′τ¯>0 when *τ* = *τ*_*j*_^+^, and Reλ′τ¯<0 when *τ* = *τ*_*j*_^−^.

**Theorem 4 .**

If $\left(m-w\right)\sqrt{\Delta }-wB<0$, then the Hopf bifurcation of system (4) at positive equilibrium *E*_3_(*x*^∗^, *y*^∗^) when *τ* = *τ*_*j*_ is supercritical (subcritical) and the bifurcating periodic solutions on the manifold are stable (unstable) if Re[*C*_1_(0)] < 0 (Re[*C*_1_(0)] > 0).

**Theorem 5 .**

If $\left(m-w\right)\sqrt{\Delta }-wB>0$, ∆_1_ > 0, and *z*_1_ + *z*_2_ = 2*p* − *r*^2^ + *s*^2^ > 0, then when *τ* = *τ*_*j*_^+^, the Hopf bifurcation of system (4) at the positive equilibrium *E*_3_(*x*^∗^, *y*^∗^) is supercritical (subcritical) and the bifurcating periodic solutions on the manifold are stable (unstable) if Re[*C*_1_(0)] < 0 (Re[*C*_1_(0)] > 0);

when *τ* = *τ*_*j*_^−^, the Hopf bifurcation of system (4) at the positive equilibrium *E*_3_(*x*^∗^, *y*^∗^) is subcritical (supercritical) and the bifurcating periodic solutions on the manifold are stable (unstable) if Re[*C*_1_(0)] < 0 (Re[*C*_1_(0)] > 0).

## 6. Numerical Simulations

In this section, some numerical simulations are carried out to support our theoretical analysis.

The article "Stability and Hopf Bifurcation Analysis of an Epidemic Model with Time Delay" was retracted in 2023. Reasons: signs of a paper mill; suspected computer-generated content; unreliable results or conclusions; concerns about the data.

There are so many different cases that only the most particular one in (3) of Theorem 7 is considered in this section. The coefficients are chosen as follows: *b* = 0.4, *d* = 0.8, *w* = 1, and *m* = 6. Then, the conditions of (3) in Theorem 7 are satisfied, where

$\left(m-w\right)\sqrt{\Delta }-wB\approx 13.166>0,{∆}_{1}\approx 0.0110067>0,\text{and}2p-r^{2}+s^{2}\approx 0.319612>0$.

By direct calculation, we have

(125) $$\begin{array}{c} x^{*}\approx 0.169906,y^{*}\approx 0.049528; \end{array}$$

and

(126) $$\begin{array}{c} \tau_{0}^{+}\approx 4.25918,\tau_{0}^{-}\approx 9.66231,\tau_{1}^{+}\approx 17.8969,\tau_{1}^{-}\approx 28.8393,\tau_{2}^{+}\approx 31.5347,\tau_{2}^{-}\approx 48.0163,\tau_{3}^{+}\approx 45.1725\cdots , \end{array}$$

where *τ*_2_^−^ > *τ*_3_^+^.

From Theorem 7, we know that the positive equilibrium *E*_3_(0.169906, 0.049528) should be asymptotically stable when *τ* ∈ [0, *τ*_0_^+^) ∪ (*τ*_0_^−^, *τ*_1_^+^) ∪ (*τ*_1_^−^, *τ*_2_^+^), and it is unstable when *τ* ∈ (*τ*_0_^+^, *τ*_0_^−^) ∪ (*τ*_1_^+^, *τ*_1_^−^) ∪ (*τ*_2_^+^, +∞). The system (4) undergoes 3 switches.

All the simulation results for *τ* in the six different intervals are in consistent with the theoretical analysis, which are shown in Figures 1–6.

## Figures and Tables

**Figure 1:** The dynamic behaviors of system (4) with *τ* = 3.8 ∈ [0, *τ*_0_^+^). (a) and (b) are the waveform plot and phase for system (4), respectively. *E*_3_(*x*^∗^, *y*^∗^) is asymptotically stable and the initial condition is (0.16, 0.1).

**Figure 2:** The dynamic behaviors of system (4) with *τ* = 4.4 ∈ (*τ*_0_^+^, *τ*_0_^−^). (a) and (b) are the waveform plot and phase for system (4), respectively. *E*_3_(*x*^∗^, *y*^∗^) is unstable with the emergence of oscillation and the initial condition is (0.18, 0.12).

**Figure 3:** The dynamic behaviors of system (4) with *τ* = 11 ∈ (*τ*_0_^−^, *τ*_1_^+^). (a) and (b) are the waveform plot and phase for system (4), respectively. *E*_3_(*x*^∗^, *y*^∗^) is asymptotically stable and the initial condition is (0.1,0.06).

**Figure 4:** The dynamic behaviors of system (4) with *τ* = 23 ∈ (*τ*_1_^+^, *τ*_1_^−^). (a) and (b) are the waveform plot and phase for system (4), respectively. *E*_3_(*x*^∗^, *y*^∗^) is unstable with the emergence of oscillation and the initial condition is (0.2, 0.2).

**Figure 5:** The dynamic behaviors of system (4) with *τ* = 30 ∈ (*τ*_1_^−^, *τ*_2_^+^). (a) and (b) are the waveform plot and phase for system (4), respectively. *E*_3_(*x*^∗^, *y*^∗^) is asymptotically stable and the initial condition is (0.15, 0.02).

**Figure 6:** The dynamic behaviors of system (4) with *τ* = 36 ∈ (*τ*_2_^+^, +∞). (a) and (b) are the waveform plot and phase for system (4), respectively. *E*_3_(*x*^∗^, *y*^∗^) is unstable with the emergence of oscillation and the initial condition is (0.15, 0.14).

The article "Stability and Hopf Bifurcation Analysis of an Epidemic Model with Time Delay" was retracted in 2023. Reasons: signs of a paper mill; suspected computer-generated content; unreliable results or conclusions; concerns about the data.

## Data Availability

The data used to support the findings of the study are included within the article.
